The article "A Broad Learning System to Predict the 28-Day Mortality of Patients Hospitalized with Community-Acquired Pneumonia: A Case-Control Study" was published in 2022. Journal: Comput Math Methods Med.

# A Broad Learning System to Predict the 28-Day Mortality of Patients Hospitalized with Community-Acquired Pneumonia: A Case-Control Study

**DOI:** 10.1155/2022/7003272

**Published:** 2022-03-04

**Authors:** Jing Yuan, Xin Liu, Wen-Feng Wang, Jing-Jing Zhang

**Affiliations:** ^1^Department of Infectious Diseases, Chifeng Municipal Hospital, Chifeng Clinical Medical School of Inner Mongolia Medical University, Chifeng 024000, China; ^2^Department of Neurosurgery, Chifeng Municipal Hospital, Chifeng Clinical Medical School of Inner Mongolia Medical University, Chifeng 024000, China; ^3^School of Science, Shanghai Institute of Technology, Shanghai 201418, China

## Abstract

This study was to conduct a model based on the broad learning system (BLS) for predicting the 28-day mortality of patients hospitalized with community-acquired pneumonia (CAP). A total of 1,210 eligible CAP cases from Chifeng Municipal Hospital were finally included in this retrospective case-control study. Random forest (RF) and an eXtreme Gradient Boosting (XGB) models were used to develop the prediction models. The data features extracted from BLS are utilized in RF and XGB models to predict the 28-day mortality of CAP patients, which established two integrated models BLS-RF and BLS-XGB. Our results showed the integrated model BLS-XGB as an efficient broad learning system (BLS) for predicting the death risk of patients, which not only performed better than the two basic models but also performed better than the integrated model BLS-RF and two well-known deep learning systems-deep neural network (DNN) and convolutional neural network (CNN). In conclusion, BLS-XGB may be recommended as an efficient model for predicting the 28-day mortality of CAP patients after hospital admission.

## 1. Introduction

Pneumonia is the most common respiratory disease [1]. Before the advent of antibiotics, pneumonia was one major killer to the human health [2]. With the advances in modern medicine, many pneumonia patients have been cured with antibiotics and adjuvant therapy, but the mortality rate remains high among the very young, the elderly, and those with compromised immune functions [3]. After the initial triage of patients with pneumonia, it is critical for emergency medical staff to assess whether these patients require hospitalization [4]. Unnecessary hospitalizations not only increase the risk of acquired infections but also drain health care resources [5]. Several pneumonia severity scales may be used to assess the severity of a patient's illness, but these scales are mainly used in the inpatients and are not suitable for emergency patients [6]. Community-acquired pneumonia (CAP) is a common infectious disease of respiratory system [7]. A deep insight into the potential factors influencing the quality of antibiotic use is essentially necessary to develop effective and targeted interventions to improve care for patients with CAP [8]. Accurate disease assessment is of great value for the initial treatment, clinical stability, and long-term prognosis [9]. Biomarkers are immune cells and immune proteins that are significantly increased in the process of microbial immunity and have auxiliary diagnostic value in the evaluation of CAP [10].

Nowadays, artificial intelligence is already used to solve emergent problems for medical engineering and particularly, for predicting CAP [11]. In order to avoid the devastating effects of the CAP on the patients' daily lives and healthcare systems and to control the further spread of this virus, we not only need to make an effective early diagnosis of infected patients through effective screening but also need to predict the risk of death in CAP patients [12, 13]. A series of models and algorithms were proposed to search for optimal hidden-layer architectures, connectivity, and training parameters for deep learning systems for predicting the CAP risk among patients with respiratory complaints, but the efficiency of these models and algorithms in predicting the death risk of patients hospitalized with CAP needs a further investigation, and meanwhile, novel approaches are quite necessary [14, 15].

Our objectives in the present studies are (1) to develop an efficient model based on the previous models and algorithms for predicting the risk of the 28-day mortality in patients hospitalized with CAP, using the random forest (RF) and eXtreme Gradient Boosting (XGB) models [16]; (2) to utilize the broad learning system (BLS) extract the features and evaluate the importance of BLS features in predicting the 28-day mortality of patients [17]; and (3) to compare the performance of the proposed model with two well-known deep learning systems-deep neural network (DNN) and convolutional neural network (CNN).

## 2. Materials and Methods

### 2.1. Study Design and Population

This was a retrospective case-control study. The information of a total of 1,397 CAP patients was collected from the Chifeng Municipal Hospital between August 2019 and December 2020. After excluding cases with age < 18 years (*n* = 58), having recently received chemotherapy (*n* = 24), advanced liver disease (*n* = 67), and the serum creatinine level > 1.5 mg/dl (*n* = 38), 1,210 eligible patients were finally included in this study. This study was approved by the Institutional Review Board (IRB) of Chifeng Municipal Hospital (approval number: no. 2019_24).

The inclusion criteria were as follows: (1) age ≥ 18 years old, (2) patients diagnosed with CAP according to Chinese Guidelines for Diagnosis and Treatment of Adult Community-acquired Pneumonia, and (3) available information of 28-day mortality or survival after hospital admission.

The exclusion criteria were (1) patients who have recently received chemotherapy, corticosteroids, or other immunosuppressants; (2) exposure to antibiotics within 14 days before entering the group; (3) patients with advanced liver disease; (4) being undergoing hemodialysis; (5) patients with serum creatinine level > 1.5 mg/dl; (6) patients with severe infection; and (7) patients with immune dysfunction.

### 2.2. Data Collection

The demographic and clinical information of CAP patients were collected, including gender, age, nationality, history of diseases (allergy, hypertension, diabetes, lung disease malignant tumor, heart failure (HF)), history of surgery, smoking, drinking, systolic blood pressure (SBP), diastolic blood pressure (DBP), respiratory rate, heart rate (HR), white blood cell (WBC) counts, red blood cell (RBC) counts, hemoglobin (Hb) level, platelet (PLT) counts, aspartate aminotransferase (AST) level, serum albumin (ALB) level, blood urea nitrogen (BUN) level, creatinine (Cr) level, blood glucose (Glu) level, porcine calcitonin (PCT) level, and C-reactive protein (CRP) level. The outcome was the 28-day mortality of patients hospitalized with CAP.

### 2.3. Establishment and Validation of the Prediction Models

All CAP patients were randomly grouped into the training and testing sets with a ratio of 6 : 4. The balance test was carried out between the two sets. Six prediction models were conducted using the training set (Figure 1). The logistic regression, RF, DNN, and CNN analyses were used to establish four models to predict the risk of 28-day mortality in patients hospitalized with CAP, respectively. All study variables entered the BLS to generate 106 features. Then, the two models (BLS-RF and BLS-XGB) based on the 106 features were established using RF and XGB analyses, respectively.  Figure 2 displayed the establishment of the BLS-RF model. The area under the curve (AUC), accuracy, sensitivity, specificity, positive predict value (PPV), and negative predict value (NPV) evaluated the predictive performance of the six models. Internal validation of the six prediction models was conducted using the testing set. Receiver operating characteristic (ROC) curves of the BLS-RF, BLS-XGB, CNN, and DNN models for predicting the 28-day mortality of CAP patients were shown in Figure 3.

DNN consists of three layers, input layer, hidden layer, and output layer. Each layer is fully connected. Using the original data as the input layer, the sample features are obtained progressively through the hidden layer, and then the features in the output layer are predicted. For deep learning processes, 30 hidden layers are used.

CNN's full name is convolutional neural network, which includes three convolutional layer for feature extraction and max pooling layer for down sampling. And Fully Connected Layer for classification^2^Features are extracted by the convolutional layer, useless features are excluded by the pooling layer, and finally features in the output layer are classified and predicted by the full connection layer. In this study, four convolutional layers, one pooling layer, and one full connection layer are adopted.

### 2.4. Statistical Analysis

The normality test for measurement data was assessed by Shapiro test. The continuous variables with normal distribution were analyzed using *T* test and expressed by mean ± standard deviation (Mean ± SD). Nonnormally distributed measurement data were analyzed by Mann–Whitney *U* test and represented by median and quartile (*M*[*Q*1, *Q*3]). Categorical data were evaluated utilizing *χ*^2^ test or Fisher's exact probability method, with the number of cases and the composition ratio (*N* (%)). All missing data were filled by random forest analysis. The sensitivity analysis was carried out. All statistical analyses were performed using Python software. *P* < 0.05 was considered as a statistical difference.

## 3. Results and Discussion

### 3.1. Characteristics of Patients Hospitalized with CAP

A total of 1,210 eligible CAP patients were finally included in this study, with the mean age of 63.58 ± 15.36 years. Of which, 120 cases suffered from death during hospitalization. All patients were randomly grouped into the training (*n* = 726) and testing (*n* = 484) sets according to 6 : 4. There were no differences in gender, age, nationality, history of diseases (allergy, hypertension, diabetes, lung disease malignant tumor, and HF), history of surgery, smoking, drinking, SBP, DBP, respiratory rate, HR, WBC counts, RBC counts, Hb level, PLT counts, AST level, ALB level, BUN level, Cr level, Glu level, PCT level, and CRP level (all *P* > 0.05). It was indicated that the data was balanced between the two sets. The characteristics of CAP patients in the training and testing sets were shown in Table 1.

### 3.2. The Predictive Performance of the Models for the 28-Day Mortality of CAP Patients

The AUC values of the BLS-RF model for predicting the 28-day mortality of CAP patients were 0.979 (95% CI: 0.963-0.996) and 0.962 (95% CI: 0.936-0.988) in the training and testing sets, respectively. The AUC values of the BLS-XGB model were 0.958 (95% CI: 0.928-0.0988) and 0.943 (95% CI: 0.905-0.980) in the training and testing sets, respectively. The AUC of DNN used in training set is 0.968 (95% CI: 0.947-0.990), and the AUC in test set is 0.907 (95% CI: 0.860-0.955). The AUC of CNN in training set was 0.980 (95% CI: 0.967-0.993), and AUC in testing set was 0.938 (95% CI: 0.910-0.966). Using the basic prediction model, the AUC of RF in the training set is 0.900 (95% CI: 0.861-0.939), and the AUC in the testing set is 0.786 (95% CI: 0.727-0.846). The AUC of logistic model was 0.832 (95% CI: 0.785-0.879) in training set and 0.714 (95% CI: 0.649-0.780) in testing set. Finally, BLS is used to learn and output features, and random forest prediction is used, as shown in Figures 3 and 4.

From the AUC, we can find that the AUC of the two training models based on BLS is similar in the testing set (*P* = 0.414). However, there was no significant difference between the AUC of DNN and CNN in the testing set (*P* = 0.270). There is no significant difference between the AUC of the two basic prediction models Logistic and Random Forest in the testing set (*P* = 0.371). The AUC of the testing set of BLS-based stochastic forest model is better than that of DNN (*P* = 0.047). The AUC of integrated models in the testing set not only is better than those of basic model RF and logistic in the testing set.

### 3.3. Importance Diagram of the BLS-Based Features

As stated in Section 2, BLS is used to learn and output features, and random forest prediction is used. Among the BLS output features, the features with the highest feature importance are the 60th, 65, 74, 9, 84, 45, 18, 102, 75, and 49 among the top 10 features with the highest model importance, BLS60 is the most important, followed by BLS65, BLS49 is the lowest, see details in Figure 4.

Machine learning analysis with text representation has been utilized in some previous studies, such as early detection of readmission risk for decision support based on clinical notes, discovering the predictive value of clinical notes, deep learning approaches in chest radiograph, and deep learning techniques on chest X-ray and CT scan [18, 19]. But a further investigation on applications in predicting the death risk of CAP among hospitalized patients with respiratory complaints is still required, and a novel approach to improve the model performance is also quite necessary [20–23].

### 3.4. Comparison for the Prediction Models

The accuracy, sensitivity, specificity, PPV, and NPV of the two prediction models are established by using BLS to learn and output features, which is a brain-inspired model [24]. And then using the random forest and XGB to extract features from BLS is the highest among all models. Hence, two integrated models BLS-RF and BLS-XGB are established. The sensitivity and NPV of the BLS − RF model using the training set are 0.970 (95% CI: 0.929-1.000) and 0.997 (95% CI: 0.992-1.000), and those using the testing set are 0.925 (95% CI: 0.853-0.996) and 0.989 (95% CI: 0.979-1.000), respectively. In the training set the accuracy specificity, and PPV of the BLS-XGB model are 0.959 (95% CI: 0.944-0.973), 0.967 (95% CI: 0.953-0.980), and 0.728 (95% CI: 0.632-0.825), respectively. In the testing set, the accuracy, specificity, and PPV of the BLS-XGB model are 0.932 (95% CI: 0.909-0.954), 0.958 (95% CI: 0.939-0.977), and 0.679 (95% CI: 0.565-0.801), as shown in Figure 5.

In Section 3.2, we utilized the BLS to construct better hidden-layer architectures and connectivity to extract the data features, and in this section, we further trained parameters in the integrated broad learning system and compare the efficiency of the integrated models with previous algorithms by performance in predicting the death risk of patients with acquired pneumonia after 28-day hospitalization.

As shown in Table 2, experimental results show that the integrated model BLS-XGB (training accuracy = 95.9%, testing accuracy = 93.2%) as an efficient BLS for predicting the death risk of patients, which not only performs better than the two basic models RF (training accuracy = 79.1%, testing accuracy = 75.6%) and the integrated model BLS-RF (training accuracy = 95.9%, testing accuracy = 93.2%) but also performs better than BLS-RF (training accuracy = 91.2%, testing accuracy = 87.2%) and two well-known deep learning systems-DNN (training accuracy = 94.1%, testing accuracy = 90.3%) and CNN (training accuracy = 93.0%, testing accuracy = 89.7%), and the competitiveness of the proposed model is further proved. Suggest the integrated model BLS-XGB as an efficient BLS for predicting the death risk of patients.

This study was to develop a prediction model for the risk of the 28-day mortality in patients hospitalized with CAP, which is essentially significant for emergent treating system in intelligent decisions for modern hospitals [24–28]. The potential engineering applications of our proposed model will not be limited to the patients hospitalized with CAP [29–32]. We used RF and XGB methods after learning the sample characteristics of the data by BLS [33–38]. This approach is novel compared to the previous studies on predicting the risk of death among CAP cases [39–43]. Accuracy of the integrated model is more than 90%, indicating a robust prediction. Our model also makes prediction according to various indicators of patients. At the same time, compared with the method of the previous basic models and other competitive models, the integrated model has significantly improved the performance accuracy in practical applications. The unresolved issues are also the main challenges in treating pneumonia is that a patient's condition can deteriorate suddenly, and therefore, the subsequent emergent treatment for saving personal patients needs a further utilization of other methods in medicine and artificial intelligence.

## 4. Conclusion

BLS offers an alternative way of learning in deep structure and in the present study, after being integrated with XGB, the experiments indicate a robust prediction for control the 28-day mortality risk of CAP patients after hospital admission. The integrated model BLS-XGB was selected as an efficient model to control the 28-day mortality of patients hospitalized with CAP. For subsequent studies, we encourage other researchers to extend potential engineering applications of our proposed model (not be limited to the patients hospitalized with CAP). Another next research priority is to find accompanied methods in medicine and artificial intelligence for the emergent treatment for saving personal patients after the death risk is predicted.

## Figures and Tables

**Figure 1:** Establishment and validation of the prediction models for the 28-day mortality of CAP patients.

**Figure 2:** Establishment of the BLS-RF model for predicting the 28-day mortality of CAP patients.

**Figure 3:** (a) ROC curves based on the integrated models. (b) ROC curves based on CNN and DNN.

**Figure 4:** Importance of model features.

**Figure 5:** Bar graphs of accuracy and NPV of the models on the training (a) and testing (b) set.

**Table 1:** The characteristics of patients hospitalized with CAP.

Variables	Total (*n* = 1210)	Testing (*n* = 484)	Training (*n* = 726)	Statistics	*P*
Gender (female), *n* (%)	475 (39.26)	185 (38.22)	290 (39.94)	*χ* ^2^ = 0.361	0.548
Age, years, mean ± SD	63.58 ± 15.36	63.86 ± 15.20	63.40 ± 15.48	*t* = 0.51	0.612
Nationality (Han), *n* (%)	1060 (87.60)	431 (89.05)	629 (86.64)	*χ* ^2^ = 1.554	0.213
Allergy (yes), *n* (%)	110 (9.09)	46 (9.50)	64 (8.82)	*χ* ^2^ = 0.167	0.683
Surgery (yes), *n* (%)	325 (26.86)	140 (28.93)	185 (25.48)	*χ* ^2^ = 1.753	0.186
Hypertension (yes), *n* (%)	480 (39.67)	205 (42.36)	275 (37.88)	*χ* ^2^ = 2.432	0.119
Diabetes (yes), *n* (%)	140 (11.57)	52 (10.74)	88 (12.12)	*χ* ^2^ = 0.538	0.463
Smoking (yes), *n* (%)	395 (32.64)	171 (35.33)	224 (30.85)	*χ* ^2^ = 2.647	0.104
Drinking (yes), *n* (%)	315 (26.03)	129 (26.65)	186 (25.62)	*χ* ^2^ = 0.161	0.688
Lung disease (yes), *n* (%)	160 (13.22)	74 (15.29)	86 (11.85)	*χ* ^2^ = 3.001	0.083
Malignant autumn, *n* (%)	50 (4.13)	23 (4.75)	27 (3.72)	*χ* ^2^ = 0.782	0.376
HF (yes), *n* (%)	35 (2.89)	15 (3.10)	20 (2.75)	*χ* ^2^ = 0.123	0.726
SBP, mmHg, mean ± SD	129.71 ± 20.07	129.50 ± 20.01	129.84 ± 20.11	*t* = −0.29	0.772
DBP, mmHg, mean ± SD	80.70 ± 13.24	80.68 ± 13.12	80.71 ± 13.33	*t* = −0.04	0.972
Respiratory rate, beats/minute, mean ± SD	20.81 ± 2.43	20.85 ± 2.52	20.77 ± 2.38	*t* = 0.55	0.579
HR, beats/minute, mean ± SD	89.56 ± 18.13	89.59 ± 18.90	89.54 ± 17.61	*t* = 0.04	0.966
WBC counts, 10^9^/L, *M*(*Q*_1_, *Q*_3_)	8.23 (6.31, 11.81)	8.46 (6.33, 11.50)	8.14 (6.26,12.02)	*Z* = 0.579	0.562
RBC counts, 10^12^/L, mean ± SD	4.29 ± 0.73	4.31 ± 0.70	4.28 ± 0.74	*t* = 0.74	0.459
Hb, g/L, mean ± SD	128.09 ± 21.78	128.98 ± 21.11	127.50 ± 22.22	*t* = 1.16	0.246
PLT counts, 10^9^/L, *M*(*Q*_1_, *Q*_3_)	244.55 (193.00, 320.30)	244.55 (195.40, 328.00)	244.55 (190.00, 314.00)	*Z* = 1.013	0.311
AST, *μ*/L, *M*(*Q*_1_, *Q*_3_)	21.61 (16.00, 33.00)	21.00 (16.00, 32.00)	22.00 (16.00, 34.00)	*Z* = −0.433	0.665
ALB, *μ*/L, mean ± SD	35.48 ± 5.84	35.67 ± 5.99	35.35 ± 5.74	*t* = 0.93	0.350
BUN, mmol/L, *M*(*Q*_1_, *Q*_3_)	5.30 (4.10, 7.30)	5.35 (4.10, 7.30)	5.20 (4.10, 7.26)	*Z* = 0.561	0.575
Cr, *μ*mol/L, mean ± SD	64.16 ± 20.92	63.28 ± 20.90	64.75 ± 20.93	*t* = −1.19	0.233
Glu, mmol/L, *M*(*Q*_1_, *Q*_3_)	5.90 (5.00, 7.26)	5.80 (4.99, 7.17)	5.99 (5.00, 7.30)	*Z* = −1.203	0.229
PCT, ug/L, *M*(*Q*_1_, *Q*_3_)	0.10 (0.05, 0.34)	0.10 (0.06, 0.31)	0.10 (0.05, 0.36)	*Z* = −0.343	0.732
CRP, mg/L, *M*(*Q*_1_, *Q*_3_)	50.20 (11.90, 114.00)	43.00 (11.50, 108.00)	54.15 (12.20, 115.00)	*Z* = −1.073	0.283
Survival state, *n* (%)				*χ* ^2^ = 0.617	0.432
Survival	1090 (90.08)	432 (89.26)	658 (90.63)		
Death	120 (9.92)	52 (10.74)	68 (9.37)		

CAP: community-acquired pneumonia; SBP: systolic blood pressure; DBP: diastolic blood pressure; HR: heart rate; WBC: white blood cell; RBC: red blood cell; Hb: hemoglobin; PLT: platelet; AST: aspartate aminotransferase; ALB: albumin; BUN: blood urea nitrogen; Cr: creatinine; Glu: blood glucose; PCT: porcine calcitonin; CRP: C-reactive protein.

**Table 2:** The predictive performance of the models for the 28-day mortality of CAP patients.

Prediction models	Accuracy	Sensitivity	Specificity	PPV	NPV
Training set					
BLS-RF	0.912 (0.891-0.932)	0.970 (0.929-1.000)	0.906 (0.884-0.928)	0.512 (0.425-0.599)	0.997 (0.992-1.000)
BLS-XGB	0.959 (0.944-0.973)	0.881 (0.803-0.958)	0.967 (0.953-0.980)	0.728 (0.632-0.825)	0.988 (0.979-0.996)
DNN	0.941 (0.924-0.958)	0.926 (0.864-0.989)	0.942 (0.924-0.960)	0.624 (0.529-0.718)	0.992 (0.985-0.999)
CNN	0.930 (0.911-0.948)	0.941 (0.885-0.997)	0.929 (0.909-0.948)	0.577 (0.485-0.668)	0.993 (0.987-1.000)
Logistic	0.789 (0.758-0.818)	0.941 (0.885-0.997)	0.774 (0.742-0.806)	0.300 (0.239-0.362)	0.992 (0.985-1.000)
RF	0.791 (0.761-0.820)	0.853 (0.769-0.937)	0.784 (0.753-0.816)	0.290 (0.227-0.353)	0.981 (0.969-0.993)
Testing set					
BLS-RF	0.872 (0.842-0.902)	0.925 (0.853-0.996)	0.865 (0.833-0.898)	0.458 (0.364-0.552)	0.989 (0.979-1.000)
BLS-XGB	0.932 (0.909-0.954)	0.717 (0.596-0.838)	0.958 (0.939-0.977)	0.679 (0.565-0.801)	0.965 (0.948-0.982)
DNN	0.903 (0.877-0.929)	0.808 (0.701-0.915)	0.914 (0.888-0.941)	0.532 (0.422-0.642)	0.975 (0.960-0.990)
CNN	0.897 (0.890-0.924)	0.769 (0.655-0.884)	0.912 (0.885-0.939)	0.513 (0.402-0.624)	0.938 (0.910-0.966)
Logistic	0.779 (0.739-0.815)	0.885 (0.798-0.971)	0.766 (0.726-0.806)	0.313 (0.238-0.388)	0.982 (0.968-0.996)
RF	0.756 (0.718-0.794)	0.615 (0.483-0.748)	0.773 (0.734-0.813)	0.246 (0.172-0.320)	0.944 (0.919-0.968)

CAP: community-acquired pneumonia; BLS: broad learning system; RF: random forest; XGB: eXtreme Gradient Boosting; DNN: deep neural network; CNN: convolutional neural network; PPV: positive predictive value; NPV: negative predictive value.

## Data Availability

The data utilized to support the findings are available from the corresponding authors upon request.
